# Circular RNA CCDC66 Improves Murine Double Minute 4 (MDM4) Expression through Targeting miR-370 in Colorectal Cancer

**DOI:** 10.1155/2022/7723995

**Published:** 2022-01-11

**Authors:** Yang Mo, Qin Lu, Qi Zhang, Jie Chen, Youming Deng, Ke Zhang, Ran Tao, Weidong Liu, Yiming Wang

**Affiliations:** ^1^Teaching and Research Section of Clinical Nursing, Xiangya Hospital of Central South University, China; ^2^State Key Laboratory of Chemo/Bio-Sensing and Chemometrics, College of Chemistry and Chemical Engineering, Hunan Provincial Key Laboratory of Biomacromolecular Chemical Biology, Hunan University, Changsha 410082, China; ^3^GeneTalks Biotech Co., Ltd., Changsha, Hunan 410000, China; ^4^Blood Transfusion Department, Zibo Central Hospital, Zibo, China; ^5^Department of Essential Surgery, Xiangya Hospital, Central South University, Changsha, Hunan 410008, China; ^6^Xiangnan University, Chenzhou, Hunan 410008, China; ^7^GeneMind Biosciences Company Limited, ShenZhen 518000, China

## Abstract

**Introduction:**

Colorectal cancer (CRC), a common digestive tract tumor that contains colon and rectal cancer, is one of the three most common cancers globally. circRNAs are involved in the occurrence and development of CRC, but the mechanism of how they participate in this process remains unclear.

**Methods:**

We adopted PCR for expression measure, CCK-8 for cell proliferation detection, Transwell for cell migration and invasion detection, and dual-luciferase reporter assays to detect the potential downstream targets of CCDC66 in CRC.

**Results:**

This study showed that circRNA CCDC66 was overexpressed in CRC tissues, and after knockdown, it inhibited the proliferation, migration, and invasion of CRC cells (RKO and HCT-116) in vitro. In addition, the dual-luciferase reporter assay showed that there was a binding site between circCCDC66 and miR-370, as well as between miR-370 and murine double minute 4 (MDM4). That is, circCCDC66 upregulated the expression of MDM4 through competitively binding to miR-370. The expression of circCCDC66 in CRC tissues was positively correlated with MDM4 and negatively correlated with miR-370.

**Conclusion:**

In summary, our results indicate that circCCDC66 is a key upregulation of CRC. circCCDC66 upregulates MDM4 through competitive binding to miR-370, thereby enhancing the metastatic ability of CRC cells and promoting the development of CRC.

## 1. Introduction

Circular RNAs (circRNAs) have only newly been widely studied, despite their discovery over 40 years ago [1]. With the rise of high-throughput sequencing technology and bioinformation, several circRNAs have been recognized as regulatory factors in cellular metabolic activity [2, 3]. As the number of studies on tumor circRNAs increases, the critical role of circRNAs has been presented in different types of cancers, lung [4, 5], breast [6], thyroid [7], brain [8], and so on [9, 10]. The circRNAs also play a crucial role in CRC development and progression. circITGA7 sponges miR-3187-3p via its miR-3187-3p targeting sites to regulate CRC progression [11]. circRNA_100290 is capable of binding to miR-516b directly and promoting migration, invasion, and proliferation of CRC cells in vitro through decreasing the expression of FZD4 [12]. circFOXO3 acts as a miR-29a-3p sponge to exhibit oncogenic activity that affects the cell cycle and cell apoptosis in prostate cancer through transcriptional upregulation of SLC25A15 [13].

CRC, a common digestive tract tumor that contains colon and rectal cancer, is one of the three most common cancers globally [14]. In 2018, new CRC cases were over 1.8 million, and 881 000 deaths occurred worldwide [15]. Given this situation, therapeutic interventions with promising biomarkers need to be developed in controlling these malignancies and relieving patient mortality. Previous studies have shown that circRNAs, including circDDX17, circRNA_100290 [12], hsa_circRNA_103809 [16], and circ_0026344 [17] have essential implications for CRC progression [18, 19]. circCCDC66 has been reported as a functional miRNA sponge in gastric cancers [20], renal carcinoma cancer, lung adenocarcinoma [21], and abdominal aortic aneurysm [22]. Therefore, we would like to resolve the secret role of circCCDC66 in CRC and further elucidate the mechanism at a molecular level.

Our study reveals that circCCDC66 could promote cell proliferation, migration, and invasion in CRC and bind to miR-370 to enhance MDM4 expression. Collectively, circCCDC66 could be regarded as a novel potential target in CRC diagnosis and treatment.

## 2. Materials and Methods

### 2.1. Human Tissue Samples

CRC patients, who underwent colorectal ectomy at Xiangya Hospital of Central South University, were the resources of colorectal tumors and matched healthy tissue. 34 pairs of both tissues were collected and preserved in an ultralow temperature freezer until the next experiment. By analysis, each tumor sample had over 80% of cancer cells. To maintain integrity and isolation, tissues were held with very close attention at -80°C during frozen sectioning. Blade washing between all samples was operated by 100% ethanol. Currently, both one tumor section and one corresponding adjacent tissue in each of the 34 subjects were dissected simultaneously, totaling 68 samples. All recruited patients had no records for any preoperative treatments that were related to chemotherapy or radiotherapy. The research protocols were approved by the Clinical Research Ethics Committee of Xiangya Hospital of Central South University. All patients had signed informed consent.

### 2.2. Cell Culture

Colorectal epithelial cell lines RKO and HCT-116 (ATCC) and one normal cell NCM460 were maintained in Dulbecco's modified Eagle's medium (DMEM; Sigma-Aldrich) supplemented with 10% fetal bovine serum (FBS; Gibco). SW620 and SW480 were maintained in RPMI-1640 medium (Sigma-Aldrich) supplemented with 10% fetal bovine serum (FBS; Gibco) and 100 U mL^−1^ antibiotic/antimycotic reagent (Invitrogen) and grown at a 37°C incubator with 5% carbon dioxide.

### 2.3. Quantitative Real-Time PCR (qRT-PCR)

TRIzol reagent (Invitrogen) was employed to isolate total RNA from tissue samples. The cDNA was synthesized according to the manufacturer's instruction of the M-MLV Reverse Transcriptase kit (Invitrogen) by using approximately 2 *μ*g of total RNA. The relative gene level was estimated by qRT-PCR using a universal SYBR Green PCR kit (Toyobo, Osaka, Japan). GAPDH and U6 were utilized as endogenous controls for mRNAs and miRNAs, respectively. The standard quantification of gene level was calculated by the 2^-*ΔΔ*Ct^ approach.

### 2.4. Cell Growth Assay

The cell proliferation of diverse groups was determined by CCK-8 assay and colony formation assay. In brief, CRC cells were seeded at approximately 2 × 10^3^ cells/well in a 96-well plate with overnight incubation. At the indicated time, each well was incubated with 10 *μ*L CCK-8 reagent (Dojindo Chemical Laboratory) for 2 h at 37°C. The absorbance was recorded in an MB-580 absorbance reader (HEALES, Shenzhen, China) at 450 nm.

As for colony formation assay *in vitro*, cells (800 cells/well) were seeded in six-well plates. The cells were cultured for approximately 10 days and fixed with 4% paraformaldehyde. After washing, the plates were air-dried and the total number of clones (>50 cells/clone) was counted.

### 2.5. Transwell Assay

The invasion assay was investigated using Transwell chambers (Costar) with polycarbonate membrane (8 mm pore size) that was coated by Matrigel (BD Biosciences). The chambers were placed in 24-well Transwell. RKO or HCT-116 cells were plated onto the upper chambers. The same protocols without Matrigel were applied for the migration assay. Medium containing 10% (V/V) FBS, regarded as a source of chemoattractant, was added into the lower chambers. After administration for 48 h at 37°C, the membrane in the upper chamber was harvested and fixed. The fixed cells were stained with 10 *μ*g/mL DAPI (Solarbio, Beijing, China) for 10 min. The cells that adhered to the adaxial surface of the membrane were enumerated by an inverted microscope (Olympus IX71).

### 2.6. Cell Fractionation Assay

Cytoplasmic and nuclear RNAs were acquired using a Cytoplasmic and Nuclear RNA Purification Kit (Norgen, Thorold, ON, Canada). Briefly, cells and tumor tissues were harvested and incubated with lysis solution on ice for 5 min. The cells were then centrifuged for 3 min at 12000 g. The supernatant was collected for cytoplasmic RNA, and the nuclear pellet was used for nuclear RNA extraction.

### 2.7. Dual-Luciferase Reporter Assay

The 3′-UTR of MDM4 and circCCDC66 harboring miR-370 binding site (MDM4-WT, circCCDC66-WT) was provided by Invitrogen and fused into the downstream of the luciferase reporter in the pmirGLO Dual-Luciferase miRNA Target Expression Vector (Promega). The negative control used the 3′-UTR containing identical flanking nucleotides of MDM4 3′-UTR and circCCDC66 and the mutated miR-370 target sequence (MDM4-MUT, circCCDC66-MUT). The dual-luciferase reporter assay was performed utilizing HCT-116 and RKO cells that transfected with miR-370 mimic or scrambled control and with the luciferase vectors mentioned above in 24-well plates. 48 h posttransfection, cells were collected for assessing the luciferase activity according to the manufacturer's direction of the Dual-Glo luciferase assay kit (Promega).

### 2.8. Statistical Analysis

The data were presented as the means ± standard deviation (SD). Comparisons between groups were analyzed using two-tailed Student's *t*-tests or one-way ANOVA. All data were performed in triplicate and implemented by SPSS 20.0 software (IBM), and *P* values < 0.05 were regarded as statistically significant.

## 3. Results

### 3.1. CRC Tissues and Cell Lines Had a High Expression of circCCDC66

To investigate whether circCCDC66 had an interrelationship with CRC, the expression of circCCDC66 in 34 paired tissues was detected. As shown in Figure 1(a), CRC tissues expressed a higher level of circCCDC66 than corresponding healthy tissues. Moreover, the expression of circCCDC66 was measured in several CRC cell lines (SW620, SW480, HCT-116, and RKO) and one normal cell. As expected, the expression of circCCDC66 in CRC cell lines was indeed higher than in normal cells (Figure 1(b)), particularly in HCT-116 and RKO.

### 3.2. The Effect of circCCDC66 on Proliferation, Migration, and Invasion of CRC Cells

To deeply study the role of CCDC66 in CRC, we first overexpressed or knocked down the level of CCDC66 in HCT-116 and RKO (Figure 1(c)). The results were detected by colony formation assays and CCK-8 assays. In both RKO and HCT-116 cells, the overexpressed CCDC66 substantially promoted cell proliferation, while circCCDC66 knockdown significantly reduced the proliferation of cells compared with the control group (Figures 1(d)–1(f)). In Transwell assays, the invasive potential of RKO and HCT-116 cells was remarkably reduced by circCCDC66 knockdown (Figures 2(a) and 2(b)), and knockdown of circCCDC66 also decreased the cell migration distance of RKO and HCT116 cells (Figures 2(c) and 2(d)). Taken together, these data suggested that circCCDC66 promoted the capacity of CRC cells to proliferate, migrate, and invade *in vitro*.

### 3.3. circCCDC66 Sponged miR-370 in the Cytoplasm of CRC Cells

To determine the involved mechanisms on how circCCDC66 was dedicated to CRC cells, the subcellular localization of circCCDC66 was dissected since the subcellular distribution of circRNA broadly impacted its function. Subcellular fractionation indicated that a more substantial proportion of circCCDC66 was located at the cytoplasm (Figure 3). Previous reports demonstrated that the majority of cytoplasmic circRNAs served as competing endogenous RNAs (ceRNAs) by competitively interacting with microRNAs. Prediction software found that miR-370 was a highly potential microRNA that binded to circCCDC66. To further investigate whether miR-370 could interact with predicted target sites in circCCDC66, the reporter vectors fusing wild type or mutant type (putative binding sites for miR-370 were mutated) circCCDC66 with luciferase were generated. As speculated, the cotransfection of the circCCDC66-WT with miR-370 mimics, but not the circCCDC66-MUT, dramatically declined luciferase activities in HCT-116 and RKO cells (Figures 4(a) and 4(b)). Besides, we found that knockdown of circCCDC66 significantly increased miR-370 expression (Figure 4(f)). Altogether, these results revealed that circCCDC66 acted as a molecular sponge for miR-370, probably promoting tumorigenesis in CRC.

### 3.4. miR-370 Regulated the Expression of MDM4

In CRC, MDM4 was reported as a mechanical downstream of miR-370. Luciferase reporter assay represented that the relative luciferase activity of MDM4-WT was uniquely alleviated by cotransfection with miR-370 mimic (Figures 4(c) and 4(d)). As Figure 4(e) show, si-CCDC66 could reduce the expression of MDM4, which indicated there was a positive correlation between CCDC66 and MDM4. Furthermore, the transcriptional and translational levels of MDM4 were markedly downregulated in the miR-370 mimic group compared with that in the negative control group, while they were also remarkably upregulated in the miR-370 inhibitor group relative to that in the inhibitor control group (Figure 4(g)). These results suggested that miR-370 could be an upstream regulator of MDM4.

### 3.5. circCCDC66 Promoted the Progression of CRC Cells via miR-370/MDM4 Axis

By transiently transfecting MDM4 siRNA or miR-370 mimics into control or circCCDC6 overexpressing HCT-116 and RKO cells, we verified the correlation between circCCDC66, miR-370, and MDM4. We found that compared with control cells, the number of clones in MDM4-siRNA or miR-370 mimics transfected cells was significantly reduced, and overexpression of circCCDC6 could partially offset this reduction (Figures 5(a) and 5(b)). Similarly, MDM4-siRNA or miR-370 mimics also reduced the migration (Figures 5(c) and 5(d)) and invasion abilities (Figures 5(e) and 5(f)) of HCT-116 and RKO cells, which was reduced by overexpression of circCCDC6.

Based on the above findings, we supposed that circCCDCC66 might promote CRC progression through miR-370/MDM4 axis. Besides, we also observed the expression of MDM4 in CRC tumors and normal tissues. It was found that MDM4 was expressed higher in CRC tumors (Figure 6). So, it was verified that CCDC66 enhanced CRC progression through the miR-370/MDM4 axis.

## 4. Discussion

*In vitro*, cellular loss-of-function experiments indicated that circCCDC66 silencing significantly suppressed the proliferation, migration, and invasion of CRC cells. circCCDC66 acted as an oncogenic circRNA in CRC tumorigenesis, revealing the potential function of circRNA in CRC occurrence and development [23]. To explore the functional mechanism of circCCDC66, we searched the potential target miRNA by luciferase experiments.

Previous studies indicate that miR-370 inhibits cancer development. For instance, Yamane et al. identify that miR-370 inhibits the proliferation of bladder cancer cells as a negative regulator of SLD5 gene expression [24]. Overexpression of miR-370 could lead to the inhibition of ovarian cancer by suppressing FOXM1 at the posttranscriptional level [25]. The present study indicated that knockdown of circCCDC66 improved miR-370 expression and led to the inhibition of CRC cell proliferation, migration, and invasion. In contrast, the reduction of miR-370 expression rescued circCCDC66 knockdown-induced inhibition of CRC cell growth. The experimental results showed that circCCDC66 promoted CRC development by sponging miR-370.

A growing amount of evidence has indicated that murine double minute 4 (MDM4), and MDM2 oncoproteins are critical negative modulators of the p53 tumor suppressor [26]. Recent studies data demonstrate that MDM4 regulates the MDM2-p53 network *in vivo*. MDM4 physiologically performs a constitutive buffer against untoward p53 function, weakening p53 activity embodies its oncogenic ability [27, 28]. According to Gembarska et al.'s report, MDM4 inhibits melanoma progression by suppressing cancer cell proliferation and metastasis and increases apoptosis via reducing p53 activity [29]. In this study, we conducted a series of experiments *in vitro*, and we found that knockdown of circCCDC66 led to miR-370 abundance and inhibition of MDM4 expression in CRC. Then, the proliferation, migration, and invasion abilities of CRC were significantly inhibited.

## 5. Conclusion

In this study, we found that the expression of circCCDC66 in CRC tissues increased. The high expression of circCCDC66 significantly promotes the proliferation, migration, and invasion of CRC cells in vitro. The present study identifies the role of circCCDC66 in sponging miR-370 and its molecular mechanism in CRC. Rescue analysis showed that circCCDC66 regulates the proliferation, migration, and invasion of CRC cells by regulating the miR-370/MDM4 pathway. In summary, the role of circCCDC66 in CRC carcinogenesis via the miR-370/MDM4 axis provides a novel insight for therapy and prevention in CRC.

## Figures and Tables

**Figure 1:** CRC tissues and cell lines had a high expression of circCCDC66. (a) The expression of CCDC66 in CRC tissues and normal tissues (*n* = 34). (b) The expression of CCDC66 in CRC cell lines and normal cells. (c) The effects of over-CCDC66 and si-CCDC66 on HCT-116 and RKO. (d) Colony formation assays were used to detect the effects of over-CCDC66 and si-CCDC66 on HCT-116 and RKO cell proliferation. (e, f) CCK-8 assays were used to detect the effects of over-CCDC66 and si-CCDC66 on HCT-116 and RKO cell proliferation. ^∗^*P* < 0.05, ^∗∗^*P* < 0.01, and ^∗∗∗^*P* < 0.001.

**Figure 2:** The effect of circCCDC66 on migration and invasion of CRC cells. (a, b) The effects of si-CCDC66 on HCT-116 and RKO cell invasion. (c, d) The effects of si-CCDC66 on HCT-116 and RKO cell migration. ^∗^*P* < 0.05.

**Figure 3:** circCCDC66 sponged miR-370 in the cytoplasm of CRC cells.

**Figure 4:** miR-370 regulated the expression of MDM4. (a, b) circCCDC66-WT dramatically declined luciferase activities in HCT-116 and RKO cells. (c, d) The relative luciferase activity of MDM4-WT was uniquely alleviated by co-transfection with miR-370 mimic. (e) There was a positive correlation between CCDC66 and MDM4. (f) Knockdown of circCCDC66 significantly increased miR-370 expression. (g) The effects of miR-370 mimic and miR-370 inhibitor on MDM4 in HCT-116 and RKO. ^∗^*P* < 0.05, ^∗∗^*P* < 0.01, and ^∗∗∗^*P* < 0.001.

**Figure 5:** circCCDC66 promoted the progression of CRC cells via the miR-370/MDM4 axis. (a, b) Compared with NC, the number of clones in MDM4-siRNA or miR-370 mimics transfected cells was significantly reduced. (c, d) MDM4-siRNA or miR-370 mimics reduced the migration in HCT-116 and RKO cells. (e, f) MDM4-siRNA or miR-370 mimics reduced the invasion in HCT-116 and RKO cells. ^∗^*P* < 0.05, ^∗∗^*P* < 0.01.

**Figure 6:** The expression of MDM4 in CRC tissues and normal tissues.

## Data Availability

All the data during the current study were available from the corresponding author on reasonable request.
